This article has been retracted.

# A20 rescues hepatocytes from apoptosis through the NF-κB signaling pathway in rats with acute liver failure

**DOI:** 10.1042/BSR20180316

**Published:** 2019-01-08

**Authors:** Ke-Zhi Li, Zhi-Yi Liao, Yu-Xuan Li, Zhi-Yong Ming, Jian-Hong Zhong, Guo-Bin Wu, Shan Huang, Yin-Ning Zhao

**Affiliations:** 1 Department of Basic Experimental Research, Affiliated Cancer Hospital of Guangxi Medical University, Nanning 530021, P.R. China; 2 The First Department of Surgery, Affiliated Wuming Hospital of Guangxi Medical University, Nanning 530199, P.R. China; 3 Department of Hepatobiliary Surgery, Affiliated Cancer Hospital of Guangxi Medical University, Nanning 530021, P.R. China

**Keywords:** A20, Acute liver failure, Hepatocyte, NF-κB signaling pathway, Proliferation, Tumor necrosis factor α-induced protein 3

## Abstract

**Background:** Acute liver failure (ALF) is a disease of acute derangements in the hepatic synthetic function with defects involving innate immune responses, which was reported to be negatively regulated by tumor necrosis factor α-induced protein 3 (A20). Herein, the present study was conducted to investigate the effects the A20 protein on the proliferation and apoptosis of hepatocytes through the nuclear factor (NF)-κB signaling pathway in the rat models simulating ALF.

**Methods:** Male Wistar rats were used to simulate ALF in the model rats. Next, the positive expression of A20 and Caspase-3 proteins was measured in liver tissues. Rat hepatocytes were separated and subjected to pyrrolidine dithiocarbamate (PDTC, inhibitor of NF-κB pathway) or A20 siRNA. Additionally, both mRNA and protein levels of A20, NF-κB, tumor necrosis factor (TNF) receptor-associated factor 6 (TRAF6), and receptor-interacting protein 1 (RIP1) were determined. Finally, we detected the hepatocyte proliferation, cell cycle entry, and apoptosis.

**Results:** ALF rats displayed a lower positive expression of A20 protein and a higher expression of Caspase-3 protein. Furthermore, A20 was down-regulated, while NF-κB, TRAF6, and RIP1 were all up-regulated in ALF rats. Notably, A20 inhibited activation of NF-κB signaling pathway. The blockade of NF-κB signaling pathway enhanced proliferation and cell cycle progression of hepatocytes, whereas inhibited apoptosis of hepatocytes. On the contrary, A20 siRNA reversed the above situation.

**Conclusion:** A20 inhibits apoptosis of hepatocytes and promotes the proliferation through the NF-κB signaling pathway in ALF rats, potentially providing new insight into the treatment of ALF.

## Introduction

Acute liver failure (ALF), due to an abrupt loss of liver function resulting from either massive or sub-massive liver necrosis in patients with a healthy liver, has found to have various causes making it difficult to identify the most accurate etiology [1]. Besides, with a high mortality rate between 60 and 90%, it classifies as a serious clinical syndrome [2]. According to its neuropathological affiliation, ALF has been characterized with having cytotoxic brain edema and biochemically, it has been characterized as showing increased brain ammonia [3]. Drug toxicity, viral hepatitis, and an indeterminate etiology might be major primary ALF causes, while multiple organ failures can be a direct result of ALF [4]. Nowadays, the survival rates of those affected by ALF are increasing; however ALF is still a life-threatening condition that has a high mortality rate [5]. Liver transplantation has been known to be a beneficial therapy, and anti-toll-like receptor 4 protein signaling has been regarded as a promising target for the treatment of ALF [6]. A previous study reported that the intracellular ubiquitin-editing protein A20 (also known as tumor necrosis factor α-induced protein 3 or TNFAIP3) promotes chronic liver inflammation and cancer by decreasing hepatocyte death [7,8]. Therefore, due to this vast collection of information, we found it to be of great importance to investigate the correlation between both A20 and ALF.

A20 has long been considered as being a potent anti-inflammatory signaling molecule that manages various intracellular signaling cascades [9]. A20 was also recognized as being an NF-κB target gene as well as encoding an ubiquitin-editing enzyme, which is important for the process of inactivating the NF-κB signaling after TNF or microbial product stimulation concludes as well as for anti-apoptosis [10]. It is reported by Shembade et al. that A20 functions when limiting the strength and duration of NF-κB signaling, were associated with many regulatory proteins, including Tax1 binding protein 1 (TAX1BP1) [11]. It is also been noted that A20 dysfunction is relative to both autoimmunity and B cell lymphoma [12]. A previous study has provided that up-regulating A20 exerts a hepato-protective effect by combining several functions, such as anti-inflammatory, antioxidant, anti-apoptotic, and pro-regenerative functions [13]. Another study identified A20 potentially increasing the hepatocyte proliferation through its decreasing of the p21 level and SOCS3 expression, which could in turn enhance IL-6/STAT3 proliferative signals as well as subsequently promote liver regeneration and injury [14]. Therefore, we intend to investigate the effects A20 has on both the proliferation and apoptosis of hepatocytes through the NF-κB signaling pathway in a rat model simulating ALF.

## Materials and methods

### Ethics statement

The study was carried out with the approval of the Ethics Committee of the Affiliated Cancer Hospital of Guangxi Medical University.

### Reagents and instruments

A total of 60 male Wistar rats (weighing between 180 and 200 g and aged 6–7 weeks old) were provided by the Laboratory Animal Center of Guangxi Medical University (Nanning, China). d-Galactosamine (D-GalN, R40326) and lipopolysaccharide (LPS, R40341) were also purchased for the present study from Sigma-Aldrich Chemical Company (St Louis, MO, U.S.A.). Horseradish peroxidase (HRP)-labeled goat anti-rabbit immunoglobulin G (IgG, H-GR0009) was also purchased from the U.S.A. Diaminobenzidine (DAB, DA1010) was purchased from Beijing Solarbio Science & Technology Co., Ltd. (Beijing, China). RNeasy Plant Mini Kit was purchased from Invitrogen Company (Carlsbad, CA, U.S.A.). Enhanced chemiluminescence (ECL, WBKLS0500) was purchased from Beijing XinZeTianYou Biotechnology Co., Ltd. (Beijing, China). Cell Counting Kit-8 (CCK-8, C0037) was purchased from Beyotime Institute of Biotechnology Co. (Shanghai, China). H-7500 transmission electron microscope was purchased from Hitachi (Tokyo, Japan). HRP-labeled streptavidin working solution (HPBIO-KT419) was purchased from HePeng (Shanghai) Biotech, Ltd. (Shanghai, China). Hematoxylin–eosin (HE, PT001) was purchased from Bogoo Biotechnology (Shanghai, China). SYBR® Premix Ex Taq™ II kit (DRR081A) was purchased from Takara Biotechnology Ltd. (Dalian, China). PrimeScript RT reagent kit (DRR037A) was purchased from Takara (Dalian, China).

### Model establishment

The rats were randomly assigned to ALF (*n*=30) and normal (*n*=30) groups. Rats had *ad libitum* access to water, but were made to fast 8 h before beginning the experiment. Rats in the controlled ALF group were intraperitoneally injected with D-GalN (800 mg/kg) and subcutaneously injected with LPS (10 μg/kg) to induce ALF. Rats in the normal group were injected with an equivalent normal saline. After administration at 2, 6, 12, 24, and 48 h, the rats underwent survival rate analysis. Next, the blood was taken out, followed by biochemical analysis of aspartate aminotransferase (AST), alanine aminotransferase (ALT), and bilirubin. At the 24 h mark following both model establishment and drug administration, the livers of mice in the two groups were separated from their bodies. Parts of the liver tissues were fixed in 10% neutral formalin and subsequently used as samples. A small part of their liver tissue was fixed in 70% ethanol for samples to be used in a flow cytometry. A small amount of their liver tissue was also fixed with 4% pentanediol in order to properly perform flow cytometry detection under a transmission electron microscope. The rest of the liver tissue was stored in a refrigerator at −80°C in liquid nitrogen for further use.

### Hematoxylin–eosin staining

The tissue block was then sliced into 5 μm sections after the tissue block was repaired. The sections were dried in an oven at 80°C for 1 h. After cooling to reach room temperature, the sections were then dehydrated in gradient alcohol, cleared in xylene, washed, stained by hematoxylin for 4 min, followed by washing, and differentiated in hydrochloric acid alcohol for 10 s. After rinsing in water for 5 min, sections were immersed in ammonia for an additional 10 min, counterstained in eosin for 2 min, dehydrated in gradient alcohol, and mounted with neutral balsam in the fuming hood. The histological changes of liver tissues following all these processes were observed under the optical microscope. The samples fixed in 10% neutral formalin were fixed for more than 24 h, dehydrated with gradient alcohol, cleared in xylene, and embedded in paraffin for further use.

### Observation of liver tissue under transmission electron microscope

The liver tissues were fixed in pentanediol (100 g/l). H-7500 transmission electron microscope was used in order to observe the changes of mitochondria, nucleus, endoplasmic reticulum, nuclear chromatin, ribosome, nuclear membrane, and possibly other parts of the ultrastructure in the hepatocyte.

### Immunohistochemistry

The formalin-fixed samples were then sliced into 3 μm sections. The sections were subsequently dried in the oven overnight at 60°C, dewaxed in xylene, washed for 3 min, added in with methanol hydrogen peroxide (97 ml methanol, 3 ml 30% hydrogen peroxide), and washed. Antigen retrieval was carried out in citrate buffer and then cooled to room temperature. The sections were then rinsed in a phosphate buffered saline (PBS), blocked in serum for 40 min at 37°C, and incubated at 4°C overnight with specific primary antibodies diluted in 0.1 M PBS (pH 7.2). After PBS washing, sections were incubated with a biotinylated secondary antibody diluted in 0.5 M Tris–HCl (pH 7.6) and incubated with HRP-labeled streptavidin at a constant temperature of 37°C for 30 min. The samples were then rinsed using PBS for 5 min, developed under DAB at room temperature, observed under a light microscope, followed by a bath under tap water in order to terminate the development. After developing, samples were immersed in distilled water for 1 min, immersed in hematoxylin for 4 min, rinsed with running water, immersed in 1% hydrochloric acid alcohol for 10 s, washed with running water, and treated with 1% ammonia for 10 min. Next, the section samples were dehydrated using gradient alcohol, cleared in xylene, and mounted with neutral balsam. PBS was used in order to replace the primary antibody as the negative control (NC).

### Reverse transcription-quantitative PCR

The total RNA was extracted from the rat liver tissue using the RNA extraction kits provided. The designed primers of A20, NF-κB, tumor necrosis factor receptor-associated factor 6 (TRAF6), and receptor-interacting protein kinase 1 (RIP1) were all synthesized by Takara (Dalian, China) (Table 1). The purpose of the total RNA was to be used as a template for reverse transcription reaction into cDNA using PrimeScript RT kits. The reaction conditions were shown to be the following: reverse transcription three times (15 min per time) at a temperature of 37°C as well as reverse transcriptase enzyme inactivation at 85°C for 5 s. A PCR method was performed, according to the instructions provided by SYBR® Premix Ex Taq™ II kit. The PCR’s reaction system went as the following: 25 μl of SYBR® Premix Ex Taq™ II (2 ×), 2 μl forward primer, 2 μl reverse primer, 1 μl ROX Reference Dye (50×), 4 μl of DNA template, 16 μl double-distilled water (ddH_2_O_2_), and finally a total volume of 50 μl. The reverse transcription-quantitative PCR (RT-qPCR) was carried out using ABI PRISM® 7300 system, with the reaction conditions listed as the following: 95°C pre-denaturation for 30 s, 40 cycles of 95°C denaturation for 5 s, 60°C annealing/extension for 30 s. Glyceraldehyde-3-phosphate dehydrogenase (GAPDH) was used as the internal reference for the RT-qPCR. The relative mRNA expressions of A20, NF-κB, RIP1, and TRAF6 in the tissues were calculated. These procedures were also applied to cells following completion of transfection.

**Table 1:** Primer sequences of related genes for reverse transcription-quantitative PCR

Primer	Sequence
A20	F: 5′-CTGCCCAGGAATGCTACAGATAC-3′
	R: 5′-GTGGAACAGCTCGGATTTCAG-3′
NF-κB	F: 5′-AACAGCAGATGGCCCATACCT-3′
	R: 5′-ACGCTGAGGTCCATCTCCTTG-3′
TRAF6	F: 5′-CTGCAAAGCCTGCATCATAA-3′
	R: 5′-GGGGACAATCCATAAGAGCA-3′
RIP1	F: 5′-ACTGCTGAAGATAGGTGCTTCAGAT-3′
	R: 5′-GTAAACGGCTTCATCTACTGACCAT-3′
GAPDH	F: 5′-ACCCAGAAGACTGTGGATGG-3′
	R: 5′-GGAGACAACCTGGTCCTCAG-3′

*Note*: F, forward; R, reverse.

### Western blot analysis

Liver tissues were then added to the liquid nitrogen, ground into a uniform fine powder, lysed, and centrifuged at a rate of 13000 rpm at 4°C for 15 min, while collecting the supernatant. After having thoroughly measured the protein concentration of each sample, the samples were adjusted using deionized water in order to make sure the loading quantity of the sample stayed consistent. Sodium dodecyl sulfate (SDS) separation gel and concentration gel (10%) were prepared. The samples were then mixed along with loading buffer, boiled for 5 min, placed in an ice bath, and centrifuged thereafter. The protein samples were added into each lane equally by employing a micropipette for electrophoresis, and were subsequently transferred onto a nitrocellulose membrane. That was followed up by the protein on the gel being moved onto the nitrocellulose membranes. The membranes were then sealed in 5% skimmed milk at 4°C overnight followed by incubation overnight with primary antibodies (1:400) of A20, NF-κB, RIP1, and TRAF6. The samples were then rinsed using PBS a total of three times at room temperature (each/5 min) and incubated along with HRP-labeled IgG (1:1000) for 1 h at 37°C. The samples were then further rinsed using PBS for an additional three times (5 min per time), with an ECL reagent coloring the membrane following the PBS rinsing. Following extraction of the reagent, the membranes were covered with a plastic wrap and observed under the X-rays, with GAPDH serving as an internal reference. The mean gray value of the target protein band in relation to the internal reference band was considered as being a relative protein level. These procedures were also applied to all cells after transfection.

### Hepatocyte culture and transfection

The rats were treated with an intraperitoneal injection of phenobarbital sodium (100 μl/100 g), and then received an additional injection to the femoral vein with 1000 μl of heparin. The rats were then perfused with a quantity 500 ml of calcium-free HEPES buffer with a perfusion rate of 30 ml/min as well as 300 ml of collagenase solution that exhibited a perfusion rate of 15 ml/min for 20 min. The HEPES buffer was used to wash the collagenase solution. The digestive cleaning solution was collected and mixed in along with 100 ml of Leibovitz L-15 culture medium. Cell suspension was filtered, followed by standing for 20 min for live cell settlement. Following the live cell settlement, kept at room temperature, cells (50 g) were washed by using a low-speed centrifugation a total of three times (40 s each time) in order to remove collagenase, damaged cells, and cells of the lung parenchyma. The cells were further collected and placed into the F12 culture medium (containing a 0.2% bovine serum albumin and 10 μg/ml insulin) and were further cultured in a 5% CO_2_ incubator at a temperature of 37°C. The medium was replaced once every 48–72 h.

Hepatocytes in the logarithmic growth phase were seeded into a 6-well plate. After cell density reached between 30 and 50%, cells were transfected according to the instructions provided by the Lipofectamine 2000 kit (Invitrogen, Carlsbad, California, U.S.A.). The Opti-MEM (250 µl, Gibco, Grand Island, NY, U.S.A.) without serum being used in order to dilute 100 pmol PDTC, A20 siRNA, A20 siRNA + PDTC, and NC with a final concentration of 50 nM, followed by incubation at room temperature for 5 min. Opti-MEM (250 µl) without serum was also used in order to dilute 5 µl Lipofectamine 2000 and incubate the cells at room temperature for 5 min. The plasmid solution and Lipofectamine solution were then mixed, incubated at room temperature for 20 min, placed in a cell culture well, and cultured at a temperature of 37°C with 5% CO_2_ for 6–8 h, with the medium being replaced by a complete medium later. Following incubation between 24 and 48 h, the cells were employed for the following experiment. As a result, hepatocytes were categorized into the control group, blank group, NC group, pyrrolidine dithiocarbamate (PDTC, NF-κB inhibitor) group, A20 siRNA group, and A20 siRNA + PDTC group. The sequence of A20 was CCGTGAACACTCAGCCTTT (RiboBio Co., Ltd., Guangdong, China).

### Cell Counting Kit-8 assay

Hepatocytes were inoculated into a 96-well plate with their proper group classifications. According to the appropriate number of plated cells, each well was added along with approximately ∼100 μl of cell suspension. The culture plate was then collected at intervals of 24, 48, and 7 h after culture and being added along with 10 μl of CCK-8 reagent (reagent: culture medium = 1:10). Then, the cells were incubated at a temperature of 37°C for up to 1–2 h. The optical density (OD) value of each well was measured at the wavelength of 450 nm by a microplate reader, with each group set up three parallel wells. This experiment was repeated further a total of three times.

### Flow cytometry

Cells were treated along with 0.25% trypsin 48 h following transfection, with the cell sample being adjusted to 1 × 10^6^ cells/ml. Cells (1 ml) were then centrifuged at a rate of 1300 rpm for 10 min following collection. Per 1 ml cells were added with 2 ml PBS, centrifuged again, fixed with a 70% pre-cold ethanol solution, and placed at 4°C overnight. During the following day, the fixed cells were rinsed two times using PBS. Cell suspension (∼100 μl) was taken (cell density was not less than 10^6^ cells/ml), filtered by 300-mesh nylon mesh, and stained by using a propidium iodide (PI, 50 mg/l) containing RNAase avoiding light for 30 min. A cell cycle was analyzed at the excitation wavelength of 488 nm using flow cytometry.

Apoptosis was detected using the Annexin V-FITC/ PI double staining technique. Cell treatment was the same as what it was during the cell cycle detection. Later, the cells were cultured in a 5% CO_2_ incubator at 37°C for 48 h and were rinsed twice by PBS followed by being centrifuged. The cells were re-suspended in a 200 μl of binding buffer, stained by 10 μl of Annexin V-FITC and 5 μl of PI, reacted for 15 min at room temperature while avoiding light, and added along with 300 μl of binding buffer. Cell apoptosis was detected by adopting a flow cytometry at an excitation wavelength of 488 nm.

### Statistical analysis

Statistical analysis was performed using the SPSS 18.0 software (IBM Corp, Armonk, NY, U.S.A.). Measurement data were expressed using the mean ± standard deviation. Comparisons between two groups were conducted by performing a *t*-test. Comparisons among multiple groups were assessed by one-way analysis of variance. *P*<0.05 was considered to be statistically significant.

## Results

### Survival rate of ALF rats gradually decreases with the increasing time of drug administration

The survival rate of rats following drug administration was detected (Figure 1A). At the 6 h mark after drug administration, rats showed decreases in feeding, drinking water, and activity. At 12 h after drug administration, rats displayed slower movement, crouching, as well as a decreased reaction to stimulation. At 24 h after drug administration, rats showed a worse condition that included tachypnea, conjunctival chemosis, complete disappearance of anti-capture ability, and a slight tremor of the limbs. At 48 h after drug administration, we approached frequent deaths of the rats with the death rate of the rats reaching 90%. The survival rate of 48 h of ALF rats was shown in Figure 1. The 30 rats in the normal group within 48 h showed no death. The mRNA and protein levels of A20 in the liver tissues at a different time (6, 12, 24, and 48 h) after model establishment were detected using RT-qPCR and Western blot analysis (Figure 1B–D). Compared with the normal rats, the ALF rats showed decreased levels of A20 at different point times (6, 12, 24, and 48 h).

**Figure 1:** Survival analysis for rats within 48 h and expression of A20 at different time points (**A**) Survival analysis within 48 h of normal rats (*n*=30) and ALF rats (*n*=30, induced by injection of D-GalN 800 mg/kg and LPS 10 μg/kg). (**B**) mRNA expression of A20 within 48 h in normal and ALF rats detected by RT-qPCR. (**C**) and (**D**) Western blot analysis for protein expression of A20 within 48 h in normal and ALF rats. The data were presented as a mean ± standard deviation, analyzed by one-way analysis of variance. *P<0.05, compared with the normal group.

Biochemical analysis of AST, ALT, and bilirubin was conducted (Table 2). In comparison with normal rats, 6 h after drug administration, the aminotransferase began to increase, at 12 h after drug administration, aminotransferase reached its peak, at 24 h after drug administration, aminotransferase started to regress in the ALF rats. The bilirubin gradually elevated during the increasing time of drug administration, and at both 12 and 24 h following drug administration, there were significant differences in the ALF rats when compared with the normal group.

**Table 2:** Biochemical analysis of AST, ALT, and bilirubin of rats in each group

Group	Number	ALT (U/l)	AST (U/l)	Bilirubin (μmol/l)
Normal	6	97.86 ± 14.56	83.84 ± 10.53	166.36 ± 23.53
ALF group 2 h	6	137.67 ± 23.32	110.35 ± 17.45	215.65 ± 36.64
ALF group 6 h	6	269.68 ± 35.43*	238.22 ± 24.56*	326.74 ± 44.51*
ALF group 12 h	6	516.47 ± 45.67*	437.36 ± 42.43*	576.47 ± 58.97*
ALF group 24 h	6	324.54 ± 56.32*	312.46 ± 35.54*	725.65 ± 67.46*

*Note*: *P<0.05, compared with the normal group; measurement data were expressed as mean ± standard deviation; the data were assessed by one-way analysis of variance; *n*=6.

### ALF rats exhibit serious pathological injury, lower positive expression rate of A20 protein, and higher positive expression rate of Caspase-3 protein

HE staining method was adopted in order to detect any pathological injury in the rats. According to our results (Figure 2A), the liver tissue in the normal rats showed a normal structure, while liver tissues in the ALF rats was damaged severely, indicating swelling, acidophilic degeneration as well as necrosis of the hepatocyte, apoptotic bodies, hemorrhage, destructed hepatic lobules, and inflammatory cell infiltration observed under a light microscope.

**Figure 2:** HE staining, ultrastructure observation, and immunohistochemistry show that ALF rats display serious pathological injury, lower positive expression rate of A20 protein, and higher that of Caspase-3 protein (**A**) Image of liver tissues in normal and ALF rats using HE staining (×200); (**B**) ultrastructure observation of hepatocytes in normal and ALF rats (×20000); (**C**) positive expression rate of A20 protein in normal and ALF rats using immunohistochemistry (×200); (**D**) positive expression rate of Caspase-3 protein in normal and ALF rats using immunohistochemistry (×200); measurement data were expressed as mean ± standard deviation; the data were assessed by *t*-test; *n*=6. ***, *P*<0.001; ****, *P*<0.0001.

Ultrastructure of the hepatocytes was observed under an H-7500 transmission electron microscope (Figure 2B). The ultrastructure of the hepatocytes in the normal rats was relatively complete, displaying a round nucleus, apparent nucleolus, evenly distributed chromatin, clear nucleus, long or spherical mitochondria with arrangement in order, clearly visible ridge with the same size, rough endoplasmic reticulum arranged in order, and a rich nuclear protein. The ultrastructure of the hepatocytes in ALF rats changed noticeably, showing obvious hepatocyte swelling, decreased microvilli, hepatocytes with a disorderly arrangement, protuberance of the nuclear membrane presenting as having an acute angle or bulge of the nuclear membrane as a sphere, highly concentrated agglutination of the nuclear chromatin with an increased electron density, concentration in the side of the nuclear membrane, uneven thickness, and finally a clearly visible cell membrane. Cells were found with multiple nucleoli. The mitochondria appeared swollen; the ridge was short with some of them disappeared, while some appear vacuolar. The rough endoplasmic reticulum had expanded throughout the present study. These findings helped to provide evidence that ALF rats show significant changes in the ultrastructure of hepatocytes.

To determine the positive expression rate of A20 protein, an immunohistochemistry was performed. The positive expression rate of the A20 protein in the normal group following immunohistochemistry was shown as being relatively higher with clearly visible hepatic lobules (Figure 2C). The positive expression rate of the A20 protein in ALF rats was displayed as relatively lower with both tissue necrosis and apoptosis being present. Meanwhile, the positive expression rate of Caspase-3 protein was lower in the normal group with clearly visible hepatic lobules, while on the contrary, it was higher in the ALF group along with tissue necrosis and apoptosis (Figure 2D). These findings revealed that the there was a lower positive expression rate of A20 protein and higher positive expression rate of the Caspase-3 protein.

### A20 is down-regulated, while NF-κB, TRAF6, and RIP1 are up-regulated in ALF rats

Both RT-qPCR and Western blot analysis methods were adopted in order to detect the mRNA and protein levels of A20, NF-κB, TRAF6, and RIP1. The results of RT-qPCR (Figure 3A) showed that when compared with the normal group, the mRNA expression showed that A20 decreased, but the mRNA expressions of NF-κB, RIP1 and TRAF6 both increased in the ALF group (all *P*<0.05). The results of the Western blot analysis (Figure 3B) revealed that in comparison with the normal group, the protein level of A20 was reduced, but the protein levels of both NF-κB and RIP1 elevated in the ALF group (all *P*<0.05). These results indicated that A20 was down-regulated, while NF-κB, TRAF6, and RIP1 were all up-regulated in ALF rats.

**Figure 3:** RT-qPCR and Western blot analysis show that A20 is down-regulated, while NF-κB, TRAF6, and RIP1 are up-regulated in ALF rats (**A**) mRNA expressions of A20, NF-κB, TRAF6, and RIP1 in liver tissues detected by RT-qPCR; (**B**) protein levels of A20, NF-κB, TRAF6, and RIP1 in liver tissues detected by Western blot analysis; (**C**) protein band patterns of A20, NF-κB, TRAF6, and RIP1 in liver tissues detected by Western blot analysis; *P<0.05, ***, *P*<0.001; ****, *P*<0.0001 compared with the normal group; measurement data were expressed as mean ± standard deviation; the data were assessed by *t*-test; *n*=6.

### A20 enhances the proliferation of hepatocytes in ALF rats

The proliferation of the hepatocytes at intervals of 0, 24, 48, and 72 h after transfection was detected by using a CCK-8 assay with the relative proliferation rate of hepatocytes being calculated soon after. Results showed that in comparison with the control group, the proliferation rate in the blank, NC, PDTC, A20 siRNA, and A20 siRNA + PDTC groups were all decreased (all *P*<0.05). When compared with both the blank and NC groups, the proliferation rate in the A20 siRNA group decreased, while the proliferation rate in the PDTC group increased (all *P*<0.05); the A20 siRNA + PDTC group showed no obvious or significant difference (*P*>0.05) (Figure 4). The results showed that A20, as a negative regulator of NF-κB, could promote the proliferation of hepatocytes in ALF rats by inhibiting the NF-κB signaling pathway.

**Figure 4:** CCK-8 assay shows that A20 promotes the proliferation of hepatocytes in ALF rats *P<0.05, compared with the control group; ^#^*P*<0.05, compared with the blank and NC groups; measurement data were expressed as mean ± standard deviation; the data at different time points were assessed by repeated-measures analysis of variance. The experiment was conducted three times independently.

### A20 promotes cell cycle progression and inhibits apoptosis of hepatocytes

Next, a PI single staining of flow cytometry was used for the detection of the cell cycle entry (Figure 5A,B). The proportions of G0/G1 stage cells in the control, blank, NC, PDTC, A20 siRNA, and A20 siRNA + PDTC groups were 47.89 ± 4.56, 73.38 ± 6.45, 71.02 ± 6.32, 59.68 ± 5.12, 84.69 ± 7.43, and 66.37 ± 5.45%, while the proportions of S stage cells in each group were 39.40 ± 3.15, 16.21 ± 2.46, 16.61 ± 2.49, 24.81 ± 3.12, 8.86 ± 1.86, and 15.98 ± 2.53%. In comparison with the control group, the blank, NC, PDTC, A20 siRNA, and A20 siRNA + PDTC groups all mainly showed that the G0/G1 stage extended (cell proportion increased) and S stage shortened (cell proportion decreased) (all *P*<0.05). When compared with those of the blank and NC groups, the PDTC group showed that the G0/G1 stage shortened (cell proportion decreased) as well as the S stage extension (cell proportion increased), however the A20 siRNA group showed that there was a G0/G1 stage extension (cell proportion increased) along with S stage shortening (cell proportion decreased) (*P*<0.05), with the A20 siRNA + PDTC group showing no obvious differences (*P*>0.05).

**Figure 5:** Flow cytometry shows that A20 promotes cell cycle progression and inhibits apoptosis of hepatocytes in ALF rats (**A**) Cell cycle entry in each group determined by PI staining of flow cytometry; (**B**) cell proportion in different stages in each group; (**C**) apoptosis of hepatocytes in each group detected by Annexin V-FITC/PI double staining of flow cytometry; (**D**) apoptotic rate of rats in each group; *P< 0.05, compared with the control group; ^#^*P*<0.05, compared with the blank and NC groups; measurement data were expressed as mean ± standard deviation; the data were assessed by one-way analysis of variance. The experiment was conducted three times independently.

Next, the cell apoptosis was detected by Annexin V-FITC/PI double staining of flow cytometry (Figure 5C,D). It showed that when compared with the control group, the hepatocyte apoptosis rate in the blank, NC, PDTC, A20 siRNA, and A20 siRNA + PDTC groups all increased significantly along with the extension of time (*P*<0.05). In comparison with both the blank and NC groups, cell apoptosis involving the A20 siRNA group was increased while the same in the PDTC group decreased (all *P*<0.05). Cell apoptosis in the A20 siRNA + PDTC group, blank group, and NC group all showed no marked differences (*P*>0.05) These results indicated that A20 could very well inhibit the activation of the NF-κB signaling pathway in hepatocytes as well as inhibit the apoptosis of hepatocytes.

### A20 inhibits activation of NF-κB signaling pathway

Again both the RT-qPCR and Western blot analysis were adopted, this time in hopes of detecting both the mRNA and protein levels of A20, NF-κB, TRAF6, and RIP1 in the hepatocytes after transfection. The results of the RT-qPCR (Figure 6A) showed that, when compared with both the blank and NC groups, there were no significant differences found in the mRNA expressions of A20, NF-κB, TRAF6, and RIP1 (*P*>0.05). In comparison with the control group, the mRNA expressions of A20 in the blank, NC, PDTC, A20 siRNA, and A20 siRNA + PDTC groups were all decreased, but the mRNA expressions of NF-κB, TRAF6, and RIP1 were increased (all *P*<0.05). In comparison along with the blank and NC groups, the expression of A20 in the PDTC group showed that it had increased, while decreased mRNA expressions of NF-κB, TRAF6, and RIP1 were manifested, however the expressions of A20 in A20 siRNA group were also decreased, with elevation in the mRNA expressions of NF-κB, TRAF6, and RIP1 (all *P*<0.05). The A20 siRNA + PDTC, blank, and NC groups showed no marked differences in these expressions (*P*>0.05).

**Figure 6:** RT-qPCR and Western blot analysis show that A20 inhibits activation of NF-κB signaling pathway in hepatocytes of ALF rats (**A**) mRNA expressions of A20, NF-κB, TRAF6, and RIP1 in hepatocytes after transfection detected by RT-qPCR; (**B**) protein levels of A20, NF-κB, TRAF6, and RIP1 in hepatocytes after transfection detected by Western blot analysis; (**C**) protein band patterns of A20, NF-κB, TRAF6, and RIP1 in hepatocytes after transfection detected by Western blot analysis; *P<0.05, compared with the control group; ^#^*P*<0.05, compared with the blank and NC groups; measurement data were expressed as mean ± standard deviation; the data were assessed by *t*-test. The experiment was conducted three times independently.

The results of the Western blot analysis (Figure 6B,C) displayed that the blank and NC groups indicated no marked difference in the protein expressions of A20, NF-κB, TRAF6, and RIP1 (*P*>0.05). When compared with those of the control group, the protein expression of A20 in the blank, NC, PDTC, A20 siRNA, and A20 siRNA + PDTC groups was reduced, but the protein expressions of NF-κB, TRAF6 and RIP1 had all increased (all *P*<0.05). In comparison with the blank and NC groups, the expression of A20 in the PDTC group showed elevation, with noticeably decreased protein expressions of NF-κB, TRAF6, and RIP1, while the expression of A20 in the A20 siRNA group was decreased, elevated protein expressions of NF-κB, TRAF6, and RIP1 were all presented (all *P*<0.05). The A20 siRNA + PDTC, blank and NC groups showed no marked differences in these expressions (*P*>0.05). These findings indicated that A20 inhibits activation of NF-κB signaling pathway.

## Discussion

ALF has been universally recognized as being a life-threatening end-stage liver disease; the etiologic factors of 19% ALF patients are still unclear, with high mortality rates between 20 and 68% among the population [15–17]. A20 (TNFAIP3) is a protein taking part in the negative feedback regulation of the NF-κB signaling in order to specify pro-inflammatory stimuli in various cell types [18]. The aim of the present study was to investigate the role A20 had through the NF-κB signaling pathway in ALF.

Initially, the data implied that ALF rats displayed that both AST and ALT showed an increase at first while decreasing soon after, with the bilirubin gradually elevating with the increasing time of drug administration. Kadowaki et al. had also revealed in his report that the levels of AST, ALT, and bilirubin in ALF rats were significantly elevated [19]. Moreover, we found that the liver tissue of the ALF rats showed serious injury, lower positive expression rate of A20 protein, higher positive expression rate of Caspase-3 protein, indicative of swelling, acidophilic degeneration and necrosis of hepatocyte, apoptotic bodies, hemorrhage, destructed hepatic lobules, and inflammatory cell infiltration. In addition, Caspase-3 is not only very important in neuronal apoptosis but also regarded as the terminal event prior to cell death [20], suggesting that a higher expression rate of Caspase-3 refers to an increased apoptosis. It has also been reported that Caspase-3-dependent cleavage of CK18 at Asp396 exposes a neo-epitope, M30, which also classifies as an apoptosis marker increased in liver injury [21,22]. Moreover, ALF has been associated with massive short-term cell death, and hepatic stellate cells (HSC) activation along with a progenitor response in ALF [23].

The present study also demonstrated that up-regulating A20 inhibited hepatocyte apoptosis while promoting proliferation in ALF. It has also been demonstrated that A20 could affect the cell cycle, immune response ability, and regulatory processes, while A20 in the liver also enriches the process of oxidoreductase and electron carrier activity, as well as the oxidation–reduction processes, indicating that A20 influences the ability of the hepatocytes via production of energy and handling of the oxidative stress [24]. Up-regulating A20 in hepatocytes plays a key role in protecting cells from apoptosis and suppressing inflammation through the inhibition of the NF-κB signaling pathway with A20 being identified as an effective gene therapy aimed at preventing and treating viral and toxic ALF [25]. Furthermore, it has been revealed that up-regulating A20 in endothelial cells could in part inhibit TNF-induced and Fas-induced apoptosis [26]. Pinna et al. suggested that increased A20 protects hepatocytes from TRAIL-induced apoptosis [27]. Furthermore, it was found that the hepatoprotective effect of A20 had been associated with the activation of the NF-κB signaling pathway during ALF. Investigation has led us to witness that the myeloid-A20-deficient mice showed high levels of inflammatory cytokines in the serum, along with sustained activation of NF-κB as well as a high production of TNF via macrophages [18]. Experiments also noted that the ALF showed high inducible nitric oxide synthase (iNOS) immunoreactivity in astrocytes, and iNOS, which makes contribution to cell swelling known to be activated by the NF-κB signaling pathway [28]. It has been noted that A20 plays a key role in the suppression of both the duration and strength of the NF-κB signaling pathway as well as of the regulatory proteins such as TAX1BP1, the E3 ubiquitin ligases Itch, and ring finger protein 11 (RNF11), which are needed for the restriction of the NF-κB signaling activation [11]. The blockade of NF-κB activation led to massive hepatocyte apoptosis [29]. And hepatocyte apoptosis correlates with active NF-κB expression and disease severity of nonalcoholic and alcoholic steatohepatitis [30]. Other evidence has demonstrated that A20 could realistically improve the outcomes in kidney disease with A20 protein exerting potent NF-κB inhibitory effects in renal proximal tubular epithelial cells, shutting down the up-regulation of pro-inflammatory molecules such as both MCP-1 and ICAM-1 [31]. Produced by activated Kupffer cells in the liver, IL-6 is one of the most important NF-κB-dependent cytokines, and expression of IL-6 has been shown to be high in liver cirrhosis as well as hepatocellular carcinoma, therefore, indicating that NF-κB in liver myeloid cells positively promotes liver cancer development through IL-6 [32].

## Conclusion

In conclusion, we discovered that the A20 protein inhibits apoptosis and promotes the proliferation of hepatocytes through the NF-κB signaling pathway, thereby alleviating ALF, which may be a new clinical target in the treatment of ALF. Recently discovered single-nucleotide polymorphisms in the A20 locus are associated with numerous autoimmune and inflammatory disorders, which highlight their clinical implication [33]. Further studies are necessary and will be conducted in the future, based on larger sample sizes and more detailed methods.

## Abbreviations

ALF: acute liver failure
ALT: alanine aminotransferase
AST: aspartate aminotransferase
A20: tumor necrosis factor α-induced protein 3
CCK-8: Cell Counting Kit-8
DAB: diaminobenzidine
D-GalN: d-galactosamine
ECL: enhanced chemiluminescence
GAPDH: glyceraldehyde-3-phosphate dehydrogenase
HE: hematoxylin–eosin
HRP: horseradish peroxidase
iNOS: inducible nitric oxide synthase
LPS: lipopolysaccharide
NC: negative control
NF: nuclear factor
PBS: phosphate buffered saline
PDTC: pyrrolidine dithiocarbamate
PI: propidium iodide
RIP1: receptor-interacting protein 1
RT-qPCR: reverse transcription-quantitative PCR
TAX1BP1: Tax1 binding protein 1
TRAF6: tumor necrosis factor receptor-associated factor 6
